# Transepidermal water loss (TEWL) and transonychial water loss (TOWL) measurements in healthy nail apparatus

**DOI:** 10.1111/srt.13851

**Published:** 2024-07-19

**Authors:** Marta Szymoniak‐Lipska, Aleksandra Dańczak‐Pazdrowska, Adam Lipski, Katarzyna Korecka, Ryszard Żaba, Adriana Polańska

**Affiliations:** ^1^ Department of Dermatology Poznań University of Medical Sciences Poznań Poland; ^2^ Department of Urology Poznań University of Medical Sciences Poznań Poland; ^3^ Department of Dermatology and Venereology Poznań University of Medical Sciences Poznań Poland

**Keywords:** nail biology, nails, TEWL, TOWL

## Abstract

**Background:**

Although non‐invasive diagnostic methods are widely used to examine the nail apparatus (NA), studies in healthy ones are scarce, and analyzes were often conducted in small groups. In the literature, there are only a few reports on TOWL measurements. The results of TEWL studies in the proximal nailfold have not been published so far.

**Materials and Methods:**

Based on a detailed interview and physical examination, 81 volunteers (40 women and 41 men) aged from 22 to 65 years were qualified for the study. In this study, the overall examination of the NA in relation to water loss was performed for the first time, regarding the hand (d, dominant; n, non‐dominant) and finger types (number, start of count from thumbs) as well as sex and age.

**Results:**

The average TEWL value in the entire group ranged from 7.53 c.u. in the finger nd4 to 11.09 c.u. in nd1. Both in the dominant and non‐dominant hand, in the entire analyzed group, and taking into account gender, weak statistically significant relationships were observed between the finger type value and TEWL (*p* < 0.05).The TEWL values were lower moving away from the thumb, The average TOWL value in the entire group ranged from 5.01 c.u. in d1 to 7.34 c.u. in d5. Both in the dominant and non‐dominant hand, in the entire analyzed group and considering gender, statistically significant relationships were observed between the type of finger and TOWL values (*p* < 0.05). The TOWL values were higher moving away from the thumb. Subsequently, the values of TOWL and TEWL did not depend on type of hand (dominant or non‐dominant), sex and age. Weak and moderate statistically significant correlations were found between TEWL and TOWL values in the entire study group and in females, as well as in selected fingers in males (d2, nd2, d3, nd3, d5, nd5) (*p* < 0.05, *r* < 0.27).

**Conclusion:**

Non‐invasive diagnostics such TEWL and TOWL measurements are useful to assess differences in structure and function between types of fingers. However, obtained results demand further studies.

## 1 INTRODUCTION

Non‐invasive diagnostics within the nail is painless, does not carry a risk of infection, scarring or oncogenic potential. These research methods are attracting interest due to their repeatability, availability and, in most cases, relatively low costs. In examining the structure and function of the nail apparatus (NA), several useful methods may be applied, including dermatoscopy (onychoscopy), measurements of transepidermal water loss (TEWL), transonychial water loss (TOWL), capillaroscopy, photoplethysmography, and high‐frequency ultrasound.^1^

The measurement of TEWL has been of interest to researchers for many years as a source of information on the function of the epidermal barrier.^2^, ^3^, ^4^, ^5^, ^6^, ^7^, ^8^ This method is used both in scientific work and for commercial purposes, both in pharmaceutical and cosmetic research. So far, many studies which have been carried out, assessed the function of the epidermal barrier, in intact and in diseased skin, and were performed in patients with atopic dermatitis or contact eczema.^9^, ^10^ However, there is no information in the literature on previously obtained TEWL measurements of the proximal NA's folds of the hands. To detect TEWL, evaporimeters with an open measuring chamber can be used. They are equipped with two pairs of sensors placed in a plastic cylinder, open at the top and bottom. The sensors measure the humidity and temperature of the air above the skin surface, and the resulting gradient determines the TEWL value. A higher TEWL value indirectly indicates damage of the epidermal barrier.

TOWL is a modification of the water loss test which measures g the air humidity gradient over the nail plate. TOWL values are often many times higher than TEWL values in the same subjects.^11^ This method requires adapting the measuring device to the surface of the nail plate,^4^ which is possible with the use of adapters that reduce the measurement opening.^12^ So far, there have been only a few publications in the literature about TOWL in healthy individuals.^4^, ^12^, ^13^, ^14^, ^15^

The main goal of our study was to estimate the differences and correlations in TEWL values within proximal nail fold, and TOWL values among volunteers grouped according to sex and age, as well as, to determine the differences between corresponding fingers in dominant and non‐dominant hand.

### 1.1 Study group

Based on a detailed interview and physical examination, 81 volunteers (40 women and 41 men) aged from 22 to 65 years were qualified for the study. The mean age of the study group was 39.77 ± 11.47 years. The average age of women was 42.1 ± 10.7 years, while the average age of men was 37.49 ± 11.87 years. There were no statistically significant differences in the age distribution between the groups (*p* = 0.056).

The inclusion criteria for the study were age of majority and ability to give informed consent. The exclusion criteria were: manicure (except nail shortening) within 4 weeks before the examination, clinically overt onychopathy, dermatoses involving NA (e.g., psoriasis, lichen planus, alopecia areata), profession or hobby causing mechanical injuries of NA, circulatory failure or respiratory failure, diabetes, history of Raynaud's phenomenon, drugs that disrupt microcirculation (e.g., beta‐blockers), autoimmune connective tissue diseases. NA affected by trauma were not assessed.

The consent to conduct the research was obtained from the Bioethics Committee of the Medical University in Poznań (Resolution No. 53/19 and Resolution No. 239/19).

## 2 METHODS

A detailed medical interview was conducted, including comorbidities. The physical examination included a clinical assessment of the NA of the hands. Washing and disinfecting hands was prohibited less than 20 min before the examination, and it was recommended not to use emollient preparations on the day of the examination.

The tests were carried out using Tewameter® TM 300 from Courage‐Khazaka (Köln, Germany), with the manufacturer's recommended reducing diaphragm (2 mm in diameter) for examining small areas (Z00812). Tewameter® TM 300 was connected to the Cutometer MPA 580 device. For the standard opening size in Tewameter® (1 cm), the measured evaporation rate values are expressed in g/h/m^2^.^16^

According to the Tewameter® manufacturer's recommendations, due to the reduction of the measuring opening, the diameter of the measuring chamber remains unchanged (1 cm), therefore the obtained values should be treated as relative. The results can be presented in conventional units (c.u.).^16^

The measuring head was placed on the proximal nail fold in the case of TEWL and on the nail plate (on the border of its proximal and middle third) in the case of TOWL. Comparable, even pressure was applied. The examination was performed by the same researcher. Twenty measurements were taken at 1‐s intervals, and then the arithmetic mean was calculated.

Acclimatization (20 min) took place in a room with a temperature of 20–24°C. TEWL and TOWL measurements were then performed.

The abbreviations in the calculations were used as follows: nd for “finger of non‐dominant hand” and d for “finger of dominant hand.” The numbers were used in order: 1‐thumb, 2‐ index finger, 3‐middle finger, 4‐ ring finger, 5‐little finger.

## 3 RESULTS

The average TEWL value in the entire group ranged from 7.53 c.u. in the finger nd4 to 11.09 c.u. in nd1, in the women's group it ranged from 7.29 c.u. in nd4 to 11.07 c.u. in d1, while in the men's group it was from 7.77 IU. in nd4 to 12.01 c.u. in sun1. Among women, the lowest TEWL value was observed on nd5 (1.80 c.u.) and the highest on d1 (24.60 c.u.). In the group of men, the lowest TEWL value was observed on nd3 (1.70 c.u.) and the highest on d5 (25.70 j.u.). Due to the condition after mechanical trauma of NA in men, the TEWL values of three thumbs (two d1s and one nd1) were not included in the analysis.

Both in the dominant and non‐dominant hand, in the entire analyzed group, and taking into account gender, weak statistically significant relationships were observed between the finger type value and TEWL (*p* < 0.05). Both in the dominant and non‐dominant hand, the TEWL value decreased within distance from the thumb (Figure 1).

**FIGURE 1:** The TEWL value in whole group decreased with distance from the thumb in both hands.

### 3.1 Results—TOWL

The average TOWL value in the entire group ranged from 5.01 c.u. in d1 to 7.34 c.u. in d5. In the females it differed from 5.22 c.u. in d1 to 7.40 c.u. in d5. In males results ranged from 4.79 c.u. in d1 to 7.28 c.u. in d5. In females, the minimum TOWL value was observed on d1 (2.70 c.u.), and the highest value (12.80 c.u.) was obtained in d5. However, in the male group, the lowest measured TOWL value was recorded on d1 (1.10 IU), and the highest value on nd3 (17.60 IU).

Due to mechanical NA trauma prior to the examination in male patients, the TOWL values of three thumbs (two d1s and one nd1) were not included in the analysis.

Both in the dominant and non‐dominant hand, in the entire analyzed group and considering gender, statistically significant relationships were observed between the type of finger and TOWL values (*p* < 0.05). In both the dominant and non‐dominant hand, the TOWL value increased within distance from the thumb (Figure 2).

**FIGURE 2:** The TOWL value in the analyzed group increased with distance from the thumb in both hands.

In the entire study group, in the groups of women and men, there were no statistically significant differences between the TOWL values of the corresponding fingers of the dominant and non‐dominant hand (*p* > 0.05), with the exception of fingers 5 in the entire study group (*p* = 0.047). TOWL in the 5th fingers had statistically significantly higher values in the dominant hand than in the non‐dominant hand.

There was no statistically significant difference in TOWL values ​​between women and men in any type of finger. For each pair of corresponding fingers *p* > 0.05.

In most NA studies, no statistically significant relationships were found between age and TOWL values (*p* > 0.05). A weak, statistically significant relationship was observed only for nd4 (*r* = 0.230, *p* = 0.043) in the group of women and in the group of men, there were no statistically significant relationships between age and TOWL values (*p* > 0.05).

### 3.2 TEWL and TOWL correlations

Weak and moderate statistically significant correlations were found between TEWL and TOWL values in the entire study group and in females, as well as in selected fingers in males (d2, nd2, d3, nd3, d5, nd5) (*p* < 0.05, *r* < 0.27) (Table 1).

**TABLE 1:** *p* and *r* values for the relationship between TEWL and TOWL in the investigated group, and depending on the gender.

Whole group										
Type of finger	d1	d2	d3	d4	d5	nd1	nd2	nd3	nd4	nd5
*r*	**0.258**	**0.493**	**0.444**	**0.410**	**0.565**	**0.291**	**0.461**	**0.333**	**0.309**	**0.616**
*p*	**0.022**	**<0.001**	**<0.001**	**<0.001**	**<0.001**	**0.009**	**<0.001**	**0.003**	**0.005**	**<0.001**

Group of women										
Type of finger	d1	d2	d3	d4	d5	nd1	nd2	nd3	nd4	nd5
*r*	**0.426**	**0.560**	**0.561**	**0.590**	**0.590**	**0.439**	**0.413**	**0.357**	**0.401**	**0.611**
*p*	**0.006**	**<0.001**	**<0.001**	**<0.001**	**<0.001**	**0.005**	**0.008**	**0.024**	**0.100**	**<0.001**

Group of men										
Type of finger	d1	d2	d3	d4	d5	nd1	nd2	nd3	nd4	nd5
*r*	0.116	**0.461**	**0.482**	0.269	**0.555**	0.189	**0.496**	**0.347**	0.240	**0.619**
*p*	0.483	**0.003**	**0.002**	0.097	**<0.001**	0.244	**0.001**	**0.028**	0.136	**<0.001**

*Note*: nd—finger of non‐dominant hand; d—number of dominant hand; number—number of finger e.g., 2 – index finger.

### 3.3 Discussion of TEWL results

Elias et al., assessed the parameters of the skin of the lower limb and abdomen in vivo, and concluded that its water permeability was not dependent on the thickness of the stratum corneum.^17^ TEWL measurements performed in animals and humans indicated that the barrier function of the epidermis did not result solely from the thickness of the epidermal components. It has been suggested that differences in chemical composition influence the water permeability of stratum corneum.^18^

In the presented study, an open‐chamber evaporimeter and a dedicated small‐area adapter ring were used to perform measurements. This is the first analysis in the literature, in which TEWL measurements of the proximal NA's folds of the hands were performed. In the entire investigated group, as well as in the group of women and men, both in the dominant and non‐dominant hand, weak, statistically significant inverse relationships were observed between the type of finger and the TEWL value. The higher number of finger from the thumb, the TEWL value decreased. This might be due to the weakening of the epidermal barrier function of the first fingers, which are more closely involved in various types of manipulation. Greater water loss was observed in the thumbs and index fingers than in less frequently used fingers, such as the ring and little fingers. The phenomenon of increased TEWL has been described many times in diseases with loss of the normal epidermal barrier.^19^, ^20^, ^21^, ^22^

The TEWL value did not depend on whether it was measured in the dominant or non‐dominant hand. There were no statistically significant differences between women and men in the TEWL values of the corresponding fingers. Therefore, it can be assumed that the TEWL value of the nail fold does not depend on gender. A different observation regarding differences in TEWL values between genders was published by Firooz et al.^23^ The study assessed biophysical parameters of the skin in eight locations (forehead, cheek, nasolabial fold, neck, forearm, dorsal, and palmar surfaces of the hand and lower limb). Researchers described the occurrence of statistically significantly higher TEWL values in men, which they explained with a greater exposure time to different weather conditions, leading to damage in the epidermal barrier.^23^

In the entire study group and in the group of women, there was no statistically significant relationship between age and TEWL value. Among men, a similar observation was made for most fingers, that is, there was no statistically significant relationship between the TEWL value and age in the group of men on d2, d3, d4, d5, nd2, nd3, nd4, nd5. However, weak, statistically significant, inverse relationships were found in d1 (*r *= 0.345, *p* = 0.034) and nd1 (*r* = −0.342, *p* = 0.036), which may be an accidental statistical finding. Although there are publications reporting a decrease in TEWL depending on age, none of them focused on measuring TEWL in the proximal NA folds of the hands. Wilhelm et al.^24^ examined TEWL using the Servo Med EP1 evaporimeter on unaffected skin in 11 anatomical areas (ankle, thigh, upper and lower back, abdomen, hand, retroauricular area, dorsal and palmar surface of the forearm, upper arm and forehead) among 14 young volunteers (7 women, 7 men; mean age 26.7 ± 2.8 years) and 15 elderly participants (7 men, 8 women, mean age 70.6 ± 13.8 years). In each of the examined areas (except for the hand and behind the ear), TEWL was statistically significantly lower in the older age group.^24^ A decrease in the TEWL value with age was also described by Ghadially et al.^25^ The measurements were performed on the skin of the forearm in a group of 6 people over 80 years of age and in a group of 15 people under 30 years of age.^25^ Another study indicating a decrease in TEWL values with age was published by Boireau‐Adamezyk et al.^26^ Forty healthy volunteers with phototypes I–III were qualified for the study. The subjects were divided into 4 groups of 10 people depending on age: G1: 18–30, G2: 30–40, G3: 40–55, and G4: 55–70 years. TEWL was measured in three locations—the face (central cheek area), relatively exposed area of the arm (dorsal surface of the arm), and relatively protected area of the arm (upper inner arm). A closed chamber evaporimeter (Vapometer; Delfin, Kuopio, Finland) was used. A linear decrease in TEWL values was demonstrated depending on age in all studied locations.^27^ Observations of the above‐mentioned researchers coincide with the results of this study in terms of TEWL measured in the nail folds of the thumbs in the group of men.

### 3.4 Discussion of TOWL results

In 1973, in vitro studies on keratinized tissues were published.^28^ The researchers determined that the water permeability through the layer obtained from the skin of the anterior abdominal wall ranged between 0.14 and 0.35 mg/cm^2^/h. Values almost ten times higher (2–3 mg/cm^2^/h) were observed when the nail plate was examined. The thickness of the stratum corneum of the epidermis consisted of 1/100 of the thickness of the nail plate. The authors suggested that the water diffusion constant was several hundred times higher in the nail than in the stratum corneum.^28^ In the 1980s, it was shown that the degree of nail hydration is one of the most important factors influencing the physical properties of the nail plate.^27^ To date, few reports have been published on the measurement of water loss within healthy NA.^4^, ^12^, ^13^, ^14^, ^15^

In the entire analyzed group, as well as in the group of women and men, both in the dominant and non‐dominant hand, weak, statistically significant relationships were observed between the TOWL value and the type of finger. The more distant finger from the thumb, the higher the TOWL value. Presumably, the nail plates of the thumb and index fingers are more exposed to the environmental factors, detergents, and disinfectants and lead to the changes occurring in the nail plates. The adaptation to unfavorable conditions which affect the water retention is more prevalent in the aforementioned fingers r than in the ring and little fingers. There were no statistically significant differences between the TOWL values of the corresponding fingers of the dominant and non‐dominant hand, except for the little fingers assessed in the entire group (*p* = 0.047). In their case, TOWL had higher values in the dominant hand, which seems to be an irrelevant statistical finding.

It was observed that TOWL values in most fingers did not depend on age. A weak statistically significant relationship was observed only for TOWL nd4 in the entire group (*r* = 0.230, *p* = 0.043), which seems to be a random statistical finding.

There were no statistically significant differences in the TOWL values of the corresponding fingers between examined females and males. Therefore, we suggest that gender did not influence the TOWL value. Similar observations regarding the lack of differences between TOWL values between women and men were made by Jemec et al.^14^ The study involved 21 volunteers, the median age was 32 years and the range was 21–71 years. The study group included 12 women and 9 men. In each volunteer, NP of one thumb was examined, without distinction between the dominant and non‐dominant hand. An open chamber evaporimeter with a 12 mm diameter opening was used. The researchers observed a statistically significant inverse relationship between age and the TOWL value (*p* < 0.018),^14^ which was not confirmed in the presented study for fingers other than nd4.

The study by Kroenauer et al.^4^ involved 10 healthy volunteers. The median age was 29 years, and the age range of the participants was 2–51 years. The publication did not provide information on the gender of the respondents. Any 4 NAs of each volunteer's hands were examined. An evaporimeter with an open measuring chamber was used for the tests. The measuring opening was sealed with plasticine. The study compared TOWL of healthy participants to TOWL of patients with onychodystrophy of various origins (fungal, psoriatic, or atopic dermatitis). Lower TOWL values, and therefore, lower water loss, were observed in the case of onychodystrophy.^4^ It is worth considering whether the lower water loss from the nail plates of the thumbs and index fingers than from the ring and little fingers may also result from changes in the structure of the nail plates and be related to subclinical onychopathy of the nail plates that are more frequently exposed to harmful factors.

A different method of measuring TOWL than in the presented study was used by Murdan et al.^15^ They tested the TOWL value using an evaporimeter with a closed condensing chamber, but similarly to the present study, using a dedicated adapter. Three people without onychopathy were recruited for the study. Hand and finger nails were analyzed. Differences in TOWL values between subjects and between fingers were assessed. TOWL values were also investigated depending on the day of measurement. The thickness of the nail plates were estimated by measuring cut nails with a micrometer.

There was a greater difference in TOWL values of finger data between different individuals than between corresponding fingers in the same individual. The authors suggested that it is more reliable to compare NAs in the same person rather than the corresponding nails in different people. In contrast to the results of this study, Murdan et al.^15^ showed a relationship between the TOWL value and the nail plate thickness, as well as differences in TOWL values in the same person in the corresponding fingers of the left and right hand and left and right foot.^15^

Similarly to the presented study, Sattler et al.^12^ did not observe statistically significant differences in TOWL values between the middle finger of the dominant and non‐dominant hand. They examined the structure and function of hand NAs using, among others, OCT and TOWL. The study included 30 healthy volunteers (24 women and 6 men) aged 19–53 years (median age 45 years). To measure TOWL, an evaporimeter with an open chamber and a mounting ring glued to the nail plate was used. OCT was used to determine the thickness of the nail plates. During the study, volunteers were asked to soak their middle finger in 38°C water for 15 min a day for the next 10 days. TOWL values were measured on the first day. The final TOWL measurements were performed on the twelfth day of the study. A return to baseline TOWL values was observed 15 min after the water bath. Daily soaking of the middle finger in water at 38°C for 15 min did not have a statistically significant effect on TOWL values measured on the twelfth day of the study.^12^

### 3.5 Discussion on the relationship between TEWL and TOWL results

In the presented study, the TOWL value was found to be higher than the TEWL value of the proximal fold of a given type of NA. This is supported by research from 2001, when TEWL values in the skin of the back of the hand and TOWL of selected NAs were compared. At that time however, the relationship between TEWL and TOWL values was not analyzed.^4^ In the presented study, in the entire group, in the group of women and in relation to d2, nd2, d3, nd3, d5, nd5 in the group of men, weak and moderate, statistically significant relationships were found between TEWL and TOWL values. The discovered relationships may suggest that with lack of conditions for measuring TOWL (e.g., plate unevenness), alternatively TEWL measurement of the proximal NP shaft can be performed. This relationship was not observed in the group of men in relation to d1, nd1, d4, and nd4. The last observation seems to be irrelevant from the point of view of the entire study group, in which the existence of a relationship between TEWL and TOWL was demonstrated and may result from the specificity of the study group of men.

The data on TEWL value measurements in the proximal NP shaft of the hands and the TOWL of the NP hands were not found in the available literature.

## 4 CONCLUSIONS

In this study the overall examination of the NA in relation to water loss was performed for the first time and featured the hand and finger types as well as sex and gender. Non‐invasive diagnostics such TEWL and TOWL measurements are useful to assess differences in structure and function between types of fingers. However, the values of TOWL and TEWL do not depend on type of hand (dominant or nondominant), sex, and age. Obtained results demand further studies.

## CONFLICT OF INTEREST STATEMENT

The authors declare no conflicts of interest.

## Data Availability

The data that support the findings of this study are available from the corresponding author upon reasonable request.
